The article "Construction of a Comprehensive Mental Health Evaluation System for Clinicians" was published in 2022. Journal: J Healthc Eng.

# Construction of a Comprehensive Mental Health Evaluation System for Clinicians

**DOI:** 10.1155/2022/7651549

**Published:** 2022-02-14

**Authors:** Wenjie Wang, Xumei Wang

**Affiliations:** Department of Psychiatry, Shengjing Hospital of China Medical University, Shenyang, China

## Abstract

**Objective:**

To detect problems of mental health disorders early and actively by constructing a comprehensive evaluation system of mental health.

**Methods:**

The evaluation system was constructed by the Minnesota personality questionnaire (MMPI), the personality questionnaire (EPQ), and the depression experience questionnaire (DEQ). Total 341 interns and residents in a general hospital were investigated with the questionnaire about psychological status, and the results were analyzed by SPSS22.0.

**Results:**

The KMO was 0.879, and the factor load of the seven factors was 0.49 to 0.856. The cumulative variance contribution reached 72.18%, and the overall consistency coefficient was 0.871. The relationship, emotional disorder, paranoia, reflection, and positive response were 0.893, 0.614, 0.867, 0.771 and 0.621, respectively. In this study, the mental health composite scores of all study subjects met a normal distribution, so level 3 scores of clinical interns and residents were established according to the deviation method.

**Conclusion:**

The constructed index system contains comprehensive indicators, good reliability efficiency, and a level 3 score, which helps individuals and hospitals to detect problems early, and provide guidance and advice for active intervention.

## 1. Introduction

Mental health problems are prevalent in every working population of the world. The Organization for Economic Cooperation and Development (OECD) study showed that about 5% and 15% of the working population in high-income countries have serious and moderate mental health problems, respectively [1]. This problem is particularly prominent for physicians, with an increasing proportion of mental illness (such as anxiety, depression, and substance abuse) [2]. For example, in the UK, 10 to 20% of doctors become depressed at some stage of their career and are at higher risk of suicide than the general population; another online survey of UK physicians found that 68% of 116 respondents were diagnosed with depression and others with bipolar disorder, anxiety, eating disorders, and substance addiction [3]. A 2014 study by researchers from the American Medical Association (AMA) and Mayo Clinic showed that 54 percent of U. S. doctors are experiencing burnout, which is higher than in other industries [4]. The suicide rate was also high, with a 40-year review study of clinicians' suicides demonstrating that male clinicians had 70% more odds of suicide than the general population and 250%–400% higher for female clinicians [5].

The article "Construction of a Comprehensive Mental Health Evaluation System for Clinicians" was published in 2022. Journal: J Healthc Eng.

Clinician mental health problems are mainly affected by the following factors: special occupational nature [6], growing working pressure, and inflexible working hours [7]. Because they know more and it is easier to access drugs, doctors are also more prone to substance addiction and abuse than the general population [8]. In addition, doctors rarely seek professional help because of the humiliation of mental illness [9].

The poor mental health state of clinicians simultaneously affects their work. Research has shown that poor mental health status will reduce the accuracy of clinical diagnosis and increase medical costs while reducing the quality of medical services that patients receive [10]. Although the mental health problems of clinicians have received wide attention, there is no relatively comprehensive evaluation method to comprehensively assess their mental health. Therefore, how to evaluate and improve the mental health of hospital clinicians has become an urgent problem for individuals, families, hospitals, and even society. As it is difficult to comprehensively evaluate the individual mental health level if the individual psychological indicators are qualified or not, this study aims to explore the comprehensive mental health evaluation method and mental health status of clinicians so as to provide a reference for early problem detection and intervention.

## 2. Materials and Methods

### 2.1. Subject Investigated

A total of 353 clinical medical interns in a third-class hospital in Shenyang with standardized training, 12 invalid questionnaires were removed, and 341 valid questionnaires were obtained, with an efficiency of 96.6%. Among them, 128 were boys (37.5%) and 213 were girls (62.5%). Among them, 18 clinical medicine interns (52.8%) and 161 residents (47.2%) conducted standardized training. The age range was 21–35 years, and the mean age was 23.2 years.

### 2.2. Selection of the Study Indicators

Using the literature analysis method, the preliminary screening indicators were discussed by the expert group of the psychiatric department of the Grade A hospital and combined with the mental health quality of Chinese adults, five psychological indicators of personality characteristics, emotion, coping mode, interpersonal relationship, and reflection function were finally established to evaluate the mental health status of doctors.

### 2.3. Source of Indicators

Data on the subjects' age, gender, and specialty were collected. The Minnesota Muhiphasic Personality Inventory (MMPI) was prepared by S. R. Hathaway and J. C. Mckinley. Song Weizhen et al. revised 566 questions, including 4 validity scales and 10 clinical scales, showing good reliability and validity of each subscale. In this study, psychopathies, paranoia, and schizophrenia 3 subscales were used as evaluation tools for personality characteristics [11].^.^

The article "Construction of a Comprehensive Mental Health Evaluation System for Clinicians" was published in 2022. Journal: J Healthc Eng.

The Eysenck Personality Questionnaire (EPQ) was prepared by J. Eysenck and revised by Liu [12]. The questionnaire has 88 questions, including 4 subscales, of which scale E measures internal and external dimension; the P scale measures neuroticism dimension; the Q scale measures psychoplasm dimension; and the L scale mainly measures the concealment of subjects. It has good reliability and validity in the Chinese population. The Q scale was used as an assessment tool for personality characteristics in this study.

#### 2.3.1. The Depression Experience Questionnaire (DEQ)

Written by Blatt et al. and revised by Liu et al. [13], the DEQ had 66 questions and a graded Likert7 score with an internal consistency coefficient of 0.65–0.79 for the five factors included in the scale and 0.81 for the full scale. The five factors of the questionnaire were significantly associated with the total score of the depression self-rating scale, and the highest correlation coefficient between self-criticism factor and SDS was 0.508, followed by the helpless factor of 0.382, the dependent factor and SDS was 0.252, the autonomy factor was 0.298, and the satisfaction factor showed a significant negative correlation with SDS of −0.148.

#### 2.3.2. State-Trait Anxiety Inventory (STAI)

Prepared by Wang [14], it is made up of subscales evaluating two different anxiety types, with a total of 40 entries. Items 1–20 are the state anxiety subscales (STAI-Form Y-I, S-AI), and items 21–40 are the trait anxiety subscales (STAI-Form Y-II, T-AI).

#### 2.3.3. Coping Style Questionnaire (CSQ)

Prepared by Xiao Plan et al., the scale consists of 62 entries with only two answers each, including six subscales with good reliability and validity, and has been widely used [15].

#### 2.3.4. Emotional-Social Loneliness Questionnaire (ESLI)

The Emotion-Social Solitude Questionnaire (ESLI) is a multidimensional questionnaire distinguishing between the four types of loneliness: emotional isolation, social isolation, emotional loneliness, and social loneliness. The ESLI contains 15 pairs of descriptions, each with four-grade scores, from 3 (usually) to 0 (rarely) [14].

#### 2.3.5. Reflective Functional Questionnaire-8 (RFQ-8)

Written by Fonagy, and revised by Xu et al. [16], it is a self-assessment tool used to assess adult reflective function. The questionnaire consisted of eight entries, a Likert7 grade score, with options from “great disagreement” to “great consent.” The score of entry 1,2,3,4,5,6 as “0,0,0,0,0,1,2,3” to form the excessive mentalization (certainty about mental states, RFQ-C) subscale; entry 2,4,5,6,8 as “3,2,1,0,0,0,0” and the entry 7 score as “0,0,0,0,1,1,2,3” to form the mentalization defect (uncertainty about mental states, RFQ-U) subscale. This study finally established five first-level psychological indicators, including personality characteristics, emotion, coping mode, interpersonal relationship, and reflective function, and 23 secondary psychological indicators, such as psychological metamorphosis, paranoia, schizophrenia, mental quality, anxiety state, and anxiety characteristics, as the mental health evaluation indicators of doctors. Index numbers are shown in Table 1.

The article "Construction of a Comprehensive Mental Health Evaluation System for Clinicians" was published in 2022. Journal: J Healthc Eng.

### 2.4. Investigation Method

The method of random group sampling was applied with clinical medical interns and standardized training residents in Shenyang. Under the unified guidance of standardized trained researchers, the students were given appropriate time to let the research subjects complete the questionnaire independently and recycle the questionnaire on the spot after filling it in.

### 2.5. Statistical Analysis

The data were entered using SPSS 22.0 software. The data were analyzed by descriptive statistical analysis, internal consistency test, and factor analysis, and the comprehensive scores of the study subjects were subjected to the normality test and the independent sample *t*-test.

## 3. Results

### 3.1. Distribution of Basic Sample Information

A total of 341 samples were collected in this study, including 180 clinical medicine interns and 161 residents with standardized training. The information distribution of the study subjects is shown in Table 2.

### 3.2. Data Standardization

#### 3.2.1. Structural Validity

Because the data is not uniform in the indicators and there are positive and reverse indicators, the original data were assimilated and normalized first. Part of the raw data are shown in Table 3.

The KMO value of this study was 0.879 (*p* < 0.01), indicating the suitability for factor analysis.

#### 3.2.2. Factor Extraction

The variance was decomposed by principal component analysis, and the resulting variable eigenvalues, variance contribution rate, and cumulative variance contribution rate are shown in Table 4. The cumulative contribution was required to be greater than 70% so that seven principal components were retained in this study. Combining the inflection point of the eigenvalue curve and the gravel diagram (scree plot, SP) of the eigenvalue (Figure 1), the figure shows from another side that the first 7 main components should be taken. To better explain the extracted factors, we maximized the orthogonal rotation of the extracted seven factors, and the eigenvalues of each factor after rotation are shown in Table 5. However, the factor load matrix obtained after rotation is shown in Table 6, indicating that the structural validity of the evaluation system in this study is good.

The article "Construction of a Comprehensive Mental Health Evaluation System for Clinicians" was published in 2022. Journal: J Healthc Eng.

#### 3.2.3. Factor Interpretation and Naming

According to the rotating factor load matrix, Factor Y1 was significantly associated with the indices X18, X19, X20, and X21; that is, Y1 is correlated with emotional loneliness and social loneliness. Factor Y1 is called a human relationship factor. Factor Y2 was significantly associated with metrices X5, X6, X7, X8, X9, and X10; that is, Factor Y2 is associated with anxiety and depression, and Factor Y2 is called an emotional dysregulation factor. Factor Y3 was significantly associated with the indices X13, X15, X16, and X17; that is Factor Y3 is associated with immature coping methods, and Factor Y3 is called a neurosis factor. Factor Y4 was significantly associated with metrices X1, X2, X3, and X4; that is, Factor Y4 is associated with severe psychotic symptoms, and Factor Y4 is called a paranoid factor. Factor Y5 was mainly significantly associated with metrices X22 and X23; that is, Factor Y5 is associated with reflective function, and Factor Y5 is called a reflective functional factor. Factor Y6 was significantly associated with metrices X12 and X14; therefore, Factor Y6 is related to problem solving and asking for help, and Factor Y6 is called an active response factor. Factor Y7 is associated with the indicator X11; that is, the factor Y7 is associated with self-satisfaction, and Factor Y7 is called a confidence factor.

### 3.3. Confidence Analysis

The internal consistency of the comprehensive evaluation system was tested, and the overall Cronbach *α* coefficient of the comprehensive mental health evaluation system was 0.871. The internal Cronbach *α* coefficient of interpersonal relationships, mood disorders, neurosis, paranoia, reflective function, and positive response to these six factors were 0.893, 0.614, 0.867, 0.771, 0.626, and 0.621, respectively, indicating the good reliability of the evaluation system.

### 3.4. The Clinician Mental Health Level 3 Score Was Established

The comprehensive scores were calculated for all study subjects and tested for normality with a Z-value of 0.044 (*p* > 0.05). Therefore, 3 all subjects scored normally distributed, and the histogram of the frequency distribution for 341 subjects is shown in Figure 2. The differences in mental health composite scores between genders and seniority were compared using independent sample *t*-tests, and the results showed that the differences in gender and seniority were not statistically significant; that is, the abovementioned factors had little impact on the mental health composite scores in this study.

The article "Construction of a Comprehensive Mental Health Evaluation System for Clinicians" was published in 2022. Journal: J Healthc Eng.

## 4. Discussion

Mental health problems are prevalent in every working population of the world [17]. It brings a great economic burden on individuals and families, but also brings huge economic losses to enterprises and society. This study completed the construction of a comprehensive evaluation system for physician mental health and was able to screen out doctors with mental health problems, contributing to early problem detection and active intervention.

In this study, we selected five psychological indicators, such as personality characteristics, emotion, coping mode, interpersonal relationship, and reflection function, and used widely used psychological measurement tools, such as the Minnesota Multiple Personality test (MMPI), the Eysenck Personality Questionnaire (EPQ), the Depression Experience Questionnaire (DEQ), and extracted psychological metamorphosis, paranoia, schizophrenia, schizophrenia, anxiety state, anxiety status, anxiety characteristics, and self-criticism as comprehensive evaluation theories [18]. A comprehensive evaluation system was built. Through the principal component analysis method, combined with the cumulative factor contribution rate, seven factors were extracted and rotated by the maximum orthogonal rotation method, which were named interpersonal factors, emotional dysregulation factors, neurosis factors, paranoid factors, reflective function factors, active response factors, and confidence factors, respectively. In study carried out by Liang [19], it is proposed that the mental health quality of Chinese adults is basically the same, indicating that the factors extracted from this study can comprehensively reflect the mental health status of individuals.

The KMO value in this study was 0.879. The factor load of the extracted factors ranged from 0.49 to 0.856. The cumulative variance contribution rate was 72.18%. It shows that the comprehensive evaluation system has a good structural validity; check the internal consistency of the comprehensive evaluation system. Among them, the overall Cronbach *α* coefficient of the comprehensive mental health evaluation system of clinicians was 0.871; the internal Cronbach of interpersonal relationships, emotional dysregulation, neurosis, paranoia, reflective function, and active response to these six factors, with coefficients of 0.893, 0.614, 0.867, 0.771, 0.626, and 0.621, respectively. It indicates that the evaluation system has a good reliability.

The article "Construction of a Comprehensive Mental Health Evaluation System for Clinicians" was published in 2022. Journal: J Healthc Eng.

On the basis of the extracted 7 factors, the comprehensive scores of 341 subjects were calculated, and the data had a statistic Z-value of 0.044 (*p* > 0.05). The scores of 341 subjects were normally distributed, and they established a level 3 score of doctors with a standard deviation as a discretization to provide the basis for individual mental health evaluation. In addition, a comparison of mental health status between genders and posts showed that the differences in gender and posts were not statistically significant. Elwer et al. [20] studies showed that when individuals engage in nonsex-dominated occupations, their mental health is negatively affected and they are also more prone to absenteeism. But studies have also shown that men's mental health is largely unaffected when pursuing nongender-dominant occupations. However, in this study, significantly more women than men were present, so gender has no effect on mental health status, a conclusion that needs to be further confirmed in future studies.

This study has certain limitations: the survey was mainly of clinical interns and residents; limited by professional, age, education, and job category; failed to explore the influence of different education and postcategories for mental health status; and the measurement of mental health should be extended to more hospitals, professionals, and posts, to confirm the utility of clinicians' comprehensive mental health evaluation system.

## 5. Conclusion

This study constructed a comprehensive evaluation system of clinicians' mental health, different from the single evaluation index, using factor analysis to evaluate the mental health from interpersonal relationship, emotion, personality characteristics, reflection function, coping mode, and self-evaluation, which comprehensively reflected the mental health status of clinicians. The evaluation system has good credibility and accuracy and can classify clinicians' mental health status, providing reference for personal identification symptoms and hospital mental health screening [18, 21].

## Figures and Tables

**Figure 1:** The inflection point of the eigenvalue curve and the gravel diagram (scree plot, SP) of the eigenvalue. Combining the inflection point of the eigenvalue curve and the gravel diagram (scree plot, SP) of the eigenvalue, the figure shows from another side that the first 7 main components should be taken.

**Figure 2:** The histogram of frequency distribution of 341 study subjects in this study. Since the subjects fit a normal distribution, the level 3 score for establishing physician mental health with a standard deviation as a discrete distance according to the discrepancy method is shown in Table 7.

The article "Construction of a Comprehensive Mental Health Evaluation System for Clinicians" was published in 2022. Journal: J Healthc Eng.

**Table 1:** Mental health evaluation indicators of physicians.

Level 1 indicators	Secondary indicators	Number
Personality characteristics	Metaphrenia	X1
	Bigoted	X2
	Split personality	X3
	Psychoticism	X4
	Anxiety state	X5
	Anxiety traits	X6
	Self-criticism	X7

Emotional state	Helplessness	X8
	Rely on	X9
	Autonomy	X10
	Satisfied	X11
	Solve the problem	X12

Coping style	Self-accusation	X13
	Turn to sb. for help	X14
	Illusion	X15
	Withdraw and keep off	X16
	Rationalization	X17
	Emotional isolation	X18
	Social isolation	X19
	Emotional loneliness	X20
	Social loneliness	X21

Reflect function	RFQC	X22
	RFQU	X23

**Table 2:** Distribution of basic information.

		Clinical intern		Chief physician	
		Example number	Percentage	Example number	Percentage
Sample		180	52.8	161	47.2
Sex	Male	70	38.9	58	36.1
	Female	110	61.1	103	63.9

**Table 3:** Standardized values for 23 index scores.

Subject investigated	1	2	3	4	5	6	7	…	341
X1	0.607	0.607	−1.498	0.607	−1.030	0.373	−0.563	…	0.841
X2	−0.624	1.500	0.286	−0.624	−1.230	−0.624	−1.534	…	1.803
X3	−0.906	−0.161	−0.906	−1.439	−1.013	−0.906	−1.119	…	2.609
X4	1.507	0.404	−0.698	−1.066	−0.698	−0.331	−0.331	…	1.874
X5	−2.037	−1.062	−1.842	−1.452	−1.355	−1.842	0.301	…	1.373
X6	−2.374	−0.699	−1.851	−2.060	−0.699	−1.327	−0.071	…	1.290
X7	−2.396	−1.782	−2.220	−1.782	−1.782	−1.255	−0.290	…	0.850
X8	−2.637	−1.960	−2.412	−0.943	−1.734	−1.621	−0.153	…	1.428
X9	−1.343	−1.118	−1.569	−0.442	−1.118	−1.794	−0.442	…	0.684
X10	1.791	1.259	1.791	1.259	1.614	1.791	1.259	…	−1.576
X11	0.405	1.208	−2.004	0.673	0.673	−1.201	0.673	…	−2.540
X12	−1.150	0.737	−0.678	−0.678	−0.206	0.266	0.737	…	0.266
X13	−1.087	−1.488	−0.687	−1.087	−1.087	−0.687	−1.087	…	2.120
X14	0.838	1.261	−0.853	−1.276	0.838	0.838	1.684	…	−0.430
X15	−1.147	−1.538	−0.756	−0.365	0.026	−1.147	−1.147	…	1.591
X16	−0.837	−2.178	−1.284	−1.284	−1.284	−1.731	−0.837	…	0.505
X17	−0.651	0.820	−0.284	−0.651	0.084	−1.387	−1.387	…	1.923
X18	−1.506	−1.506	−0.625	−0.625	0.036	−0.625	−1.506	…	1.578
X19	−1.207	−0.721	−0.721	−0.964	0.250	0.007	−1.207	…	1.221
X20	−1.101	−1.101	−0.371	−0.736	−0.188	−0.371	−1.101	…	1.639
X21	−1.118	−0.860	−0.603	−1.118	−0.345	−0.088	−1.118	…	2.488
X22	−1.193	−0.246	−2.376	−2.376	0.701	0.228	1.174	…	0.938
X23	−1.122	−0.380	−1.122	−1.122	−0.010	0.732	−1.122	…	−0.010

**Table 4:** Main component analysis table.

Initial eigenvalue				Extract the sum of the square to load		
Element	Amount to	% of the variance	Accumulate (%)	Amount to	% of the variance	Accumulate (%)
1	7.667	33.336	33.336	7.667	33.336	33.336
2	2.397	10.420	43.756	2.397	10.420	43.756
3	1.765	7.672	51.429	1.765	7.672	51.429
4	1.413	6.146	57.575	1.413	6.146	57.575
5	1.236	5.372	62.947	1.236	5.372	62.947
6	1.209	5.255	68.201	1.209	5.255	68.201
7	0.915	3.978	72.180	0.915	3.978	72.180
8	0.797	3.467	75.647			
9	0.739	3.215	78.862			
10	0.629	2.736	81.597			
11	0.509	2.213	83.810			
12	0.468	2.035	85.845			
13	0.442	1.921	87.766			
14	0.403	1.754	89.520			
15	0.363	1.580	91.100			
16	0.344	1.494	92.594			
17	0.338	1.470	94.064			
18	0.321	1.397	95.461			
19	0.270	1.175	96.636			
20	0.252	1.096	97.731			
21	0.210	0.915	98.646			
22	0.202	0.876	99.522			
23	0.110	0.478	100.000			

The article "Construction of a Comprehensive Mental Health Evaluation System for Clinicians" was published in 2022. Journal: J Healthc Eng.

**Table 5:** The rotational extraction factors are presented.

Factor	Eigenvalue	% of the variance	Accumulative total (%)
Y1	3.268	14.209	14.209
Y2	3.236	14.072	28.281
Y3	3.027	13.162	41.443
Y4	2.279	9.909	51.352
Y5	2.113	9.186	60.538
Y6	1.545	6.718	67.256
Y7	1.132	4.924	72.180

**Table 6:** Factor load matrix after rotation.

Variable	After rotation						
	Y1	Y2	Y3	Y4	Y5	Y6	Y7
X1	0.09	0.20	0.06	0.82	0.07	−0.03	0.12
X2	0.16	0.14	0.09	0.81	−0.01	−0.04	−0.18
X3	0.32	0.38	0.24	0.56	0.28	0.11	0.05
X4	0.18	0.13	0.14	0.51	0.18	0.23	0.36
X5	0.09	0.83	0.21	0.22	−0.09	0.20	−0.05
X6	0.12	0.82	0.20	0.23	−0.01	0.19	−0.05
X7	0.28	0.67	0.24	0.19	0.38	0.10	−0.04
X8	0.16	0.62	0.25	0.08	0.46	−0.10	−0.08
X9	0.21	0.49	0.21	0.06	0.25	−0.31	0.37
X10	−0.16	−0.51	−0.06	−0.14	−0.47	0.24	0.01
X11	0.04	−0.11	−0.02	0.01	−0.08	0.16	0.83
X12	0.14	0.19	−0.10	0.08	0.29	0.74	0.16
X13	0.16	0.28	0.75	0.19	0.15	0.05	−0.02
X14	0.28	0.02	−0.03	−0.01	−0.05	0.75	0.07
X15	0.10	0.22	0.80	0.09	0.23	−0.03	−0.05
X16	0.17	0.21	0.82	−0.01	0.09	−0.07	−0.09
X17	0.14	0.03	0.82	0.11	0.02	−0.07	0.18
X18	0.82	0.18	0.07	0.11	0.11	0.07	0.00
X19	0.86	0.07	0.12	0.06	0.00	0.15	0.09
X20	0.81	0.20	0.15	0.21	0.14	0.14	0.07
X21	0.80	0.09	0.22	0.14	0.07	0.09	−0.02
X22	0.01	0.12	0.18	−0.07	0.74	0.16	0.09
X23	0.15	0.03	0.13	0.28	0.77	0.05	−0.15

**Table 7:** Level 3 scoring criteria for physician mental health.

Grade	Range	Same as	Preferably
Standard	≥M + S	M − S∼M + S	≤M − S
Standard mark standardized score	≥23.462	−23.461∼23.462	≤−23.461

*Note.* M is the mean number, and S is the standard deviation.

## Data Availability

The data used to support this study are available from the corresponding author upon request.
